# A parallel randomized controlled trial examining the effects of rhythmic sensory stimulation on fibromyalgia symptoms

**DOI:** 10.1371/journal.pone.0212021

**Published:** 2019-03-01

**Authors:** Thenille Braun Janzen, Denise Paneduro, Larry Picard, Allan Gordon, Lee R. Bartel

**Affiliations:** 1 Music and Health Research Collaboratory, Faculty of Music, University of Toronto, Toronto, Ontario, Canada; 2 Wasser Pain Management Centre, Sinai Health System, Toronto, Ontario, Canada; 3 Faculty of Music, University of Toronto, Toronto, Ontario, Canada; University of Regensburg, GERMANY

## Abstract

This double-blind, two-arm parallel randomized controlled trial investigated the effects of gamma-frequency rhythmic sensory stimulation on fibromyalgia. We were interested in whether rhythmic sensory stimulation would promote significant changes in fibromyalgia and associated symptoms, and whether treatment effects would differ between two distinct treatment parameters. Fifty patients with a formal diagnosis of fibromyalgia were randomly assigned to two test groups. One group received vibrotactile stimulation from a continuous sine wave single-frequency stimulation (40 Hz) for 30 minutes, five days per week, over five weeks, concomitant with usual care. The second group completed the same treatment protocol but received a different stimulation, consisting of random and intermittent complex wave gamma-range vibrotactile stimulation. Fibromyalgia symptoms, pain severity and interference, depression symptoms, quality of life and sleep quality were assessed at baseline and post-intervention. Results indicated that there were statistically significant changes from baseline to post-treatment in measures of fibromyalgia symptom severity, pain interference, depression, and sleep quality. However, treatment outcomes did not differ significantly between groups. These findings provide preliminary evidence that gamma-frequency rhythmic vibroacoustic stimulation may decrease fibromyalgia symptoms and ease associated comorbidities, opening new avenues for further investigation of the effects of rhythmic sensory stimulation on chronic pain conditions.

## Introduction

Fibromyalgia is a pain syndrome characterized by chronic widespread pain for which no cause can be identified (e.g., tissue damage or inflammation) [1,2]. Symptomatology often includes chronic fatigue, sleep disturbance, decrements in physical functioning, and disruptions in psychological functioning such as anxiety, mood disturbances, memory problems, and lack of well-being [1–3]. According to recent population-based estimations, the prevalence of fibromyalgia in the general population ranges from 2% to 8%, with a significant female predominance [1,4]. Due to the chronic nature of the disorder, fibromyalgia symptoms can significantly impact patients’ quality of life and impose high direct and indirect medical costs, which are largely associated with treatment costs [3,5,6]. Conventional treatments for fibromyalgia are typically centered on pharmacological therapies, however, studies have found that medication alone produces only modest and short-lived results, and may cause intolerable side effects [7–14]. Consequently, complementary and alternative medical treatments have become an integral component of multi-disciplinary treatment approaches for fibromyalgia, as shown by recent studies revealing that 60-90% of patients in North America seek complementary treatment options [15–20]. Therefore, there is an urgent need to develop, investigate, and validate non-pharmacological complementary treatments to help patients manage fibromyalgia.

Vibratory analgesia is a well-described phenomenon whereby sensory stimulation delivered to the skin can reduce pain [21–25]. Mechano-acoustic vibrations have been extensively used to address acute pain during orthodontic [26–28] and cosmetic procedures [29], and is a well-established technique in orthopedic practice [30] and physiotherapy to reduce muscle soreness [31–33], low back pain [34], and orofacial pain [35]. However, little is known regarding the application of vibroacoustic stimulation in the treatment of chronic pain conditions. Previous clinical studies have explored the use of rhythmic sensory stimulation to treat fibromyalgia [36–38]. Rhythmic sensory stimulation (RSS) broadly refers to the use of sensory events - including vibrotactile, auditory, and visual flickering stimuli - applied in pulsed forms with repeated short, transient stimulus events at regular intervals, or in continuous forms which generate oscillating (e.g., sinusoidal) stimulus patterns [39]. In the context of chronic pain research, the terms vibroacoustic therapy [40–42], physioacoustic therapy [43], musically fluctuating vibrations [37], and low-frequency sound stimulation [38], are often used interchangeably to refer to the use of rhythmic gamma-frequency (30 – 120 Hz) acoustic-driven stimulation of mechanoreceptors in the body by means of chairs or beds fitted with low-frequency transducers. Chesky et al. [37] reported that fibromyalgia symptoms significantly changed after a single 30-minute treatment session, however, no significant differences were noted between whole-body stimulation with gamma-range vibroacoustic stimuli (60-100 Hz) and whole-body 20 Hz stimulation. Naghdi and colleagues [38] found that pain severity, sleep quality, and fibromyalgia severity significantly improved after ten sessions of whole-body 40 Hz RSS, however, no comparison group was included in this pilot study. In Weber et al. [36], fibromyalgia patients were randomly allocated to 4 groups: 3 experimental groups and one control group. As experimental conditions, one group received vibratory stimulation ranging from 32 – 64 Hz to five specific points of the body, while patients in the other groups listened to either classical music or received a combination of both music listening and vibroacoustic stimulation. The results of this study indicated that patients in all groups had a statistically significant change from baseline in fibromyalgia outcome measures, including the control group who did not receive any form of stimulation.

Although there are some indications that RSS may improve fibromyalgia symptoms, the few studies conducted to date have used widely differing parameters of stimulation in relation to frequencies, stimuli waveforms (sine wave vs. complex wave), temporal pattern (continuous vs. intermittent), and application protocols (whole-body vs. localized), warranting further investigation. Therefore, the present study investigated the effects of gamma frequency vibrotactile RSS on fibromyalgia symptom severity by addressing two research questions. The first question relates to the effects of different parameters of stimulation (stimuli frequency, waveform, temporal pattern). We were interested in whether treatment effects would differ between treatment parameters. To assess this question we assigned participants to two groups. One group received continuous sine wave single-frequency stimulation (40 Hz) for 30 minutes, five days per week, over five weeks, concomitant with usual care. The stimulation delivered to the second group consisted of random and intermittent complex wave gamma-range RSS with peaks at 33 Hz and 45 Hz. The second research question addresses the effectiveness of RSS to reduce fibromyalgia symptom severity.

## Materials and methods

This two-arm parallel randomized controlled trial was conducted in collaboration between the Sinai Health System and the University of Toronto (Toronto/Canada), between October 2015 and December 2016. All procedures were approved by the Mount Sinai Hospital Research Ethics Board (15-0140-E) and the Office of Research Ethics at the University of Toronto (31916) and registered at ClinicalTrials.Gov (NCT02493348). All participants provided written informed consent prior to enrolment.

### Participants

Participants were outpatients aged 18-70 years of age, with a formal diagnosis of fibromyalgia, recruited through referrals from general practitioners, rheumatologists, and neurologists from clinics and hospitals in the Greater Toronto Area (Canada). Study inclusion criteria also comprised self-reported satisfactory hearing bilaterally, ability to operate the treatment device, and ability to read and write in English. Study exclusion criteria included: acute and active inflammatory conditions (e.g., rheumatoid arthritis, osteoarthritis, autoimmune disease); unstable medical or psychiatric illness; history of epilepsy, seizures, or psychosis; pregnancy or lactation; hemorrhaging or active bleeding; thrombosis or angina pectoris; heart conditions such as hypotension, arrhythmia, pacemaker; substance abuse in the last year; prolapsed vertebral disc; and recent (past 6 months) back or neck injuries. Study eligibility criteria were pre-assessed by the referring doctor and confirmed by the study doctor or a trained researcher prior to enrollment. All participants were informed of the study design and the randomization procedure, and no suggestion was made about the superiority of either treatment.

### Interventions

Participants enrolled in the study were randomly assigned to one of two study arms (Fig 1). Both groups received 25 sessions of 30-minute rhythmic sensory stimulation over five weeks concomitant with usual care. Group one received vibrotactile stimulation from a continuous single-frequency sine wave at 40 Hz that was amplitude modulated on an 11-second cycle plus isochronous auditory stimulation with a 160 Hz tone amplitude modulated at 40Hz. Group two received vibrotactile stimulation from randomly intermittent sounds consisting of complex wave gamma-range noise with pitch peaks at 33 Hz and 45 Hz. In the initial trial study protocol, the stimulation delivered to group two was intended as a sham stimulation, however, careful spectral analysis of the stimulus conducted after study completion revealed that this was not the case. The stimulation was delivered via a portable consumer device (Sound Oasis Vibroacoustic Therapy System VTS-1000) with a built-in low-frequency transducer located at the middle back region and stereo speakers located at ear level. Participants experienced the stimulus as a mild vibrotactile sensation around the lower-back and shoulder/head area as well as a low-level hum. The vibroacoustic stimulation device was provided to participants for the duration of the study, and all 25 sessions were self-administered and completed at the patients’ homes. Participants were instructed to place the device on a comfortable chair or bed and relax. There were no restrictions regarding the type of activities participants could undertake during the 30-minute session (e.g., reading, browsing the internet). Potential unintended effects associated with the intervention, such as feeling a tingling sensation, an urgency to relieve bowel, neck discomfort due to vibration in the shoulder area, were asked to be reported in the treatment log. Participants were instructed to complete a treatment log after each session containing information regarding the time and duration of the session, any activities performed during the sessions, as well as the device settings for the volume of the auditory stimulation and the intensity of the vibrotactile stimulation. The recommended stimulation intensity corresponded to level 15 of the device (ranging from 10 to 20) for both the auditory and vibratory stimuli but could be adjusted to a comfortable level if needed. The treatment log also included an 11-point Likert scale regarding pain levels before and after each session (ranging from 0: no pain to 10: extreme pain). Study compliance was assessed at weeks 2-4 via phone or e-mail communication as well as through the treatment logs submitted at the post-intervention visit. All patients received usual care during the study.

**Fig 1:** Flowchart of study participants.

### Stimuli

The sound stimulus delivered to group one consisted of a continuous single-frequency sine wave at 40 Hz that was amplitude modulated on an 11-second cycle, plus isochronous auditory stimulation with a 160 Hz tone amplitude modulated at 40 Hz with secondary pitch peaks at 120 Hz and 200 Hz (Fig 2). The track has a 1-second fade-in and a 13-second fade-out, with an output level of -12.7db. The track features an automated volume adjustment where the first 5.5 seconds the volume decays from 2.73db to -8db, and during the second 5.5 seconds the volume increased from -8.db back to 2.73db, thus creating an on-going jig saw volume contour. The sine wave was generated using ToneGen software (NCH Software) and was recorded at 40K and 24 bit-rate into Cubase Studio 5 (Steinberg) through an M-Audio 2626 interface.

**Fig 2:** Stimulus peak frequencies. Sound stimulus delivered to group one consisted of continuous single-frequency sine wave with peak frequency at 40 Hz that was amplitude modulated on an 11-second cycle (top figure), plus isochronous auditory stimulation with a 160 Hz tone amplitude modulated at 40 Hz with secondary pitch peaks at 120 Hz and 200 Hz (bottom figure).

The second track, administered as stimulation to group two, comprised of randomly intermittent sounds consisting of complex wave gamma-range noise with pitch peaks at approximately 33 Hz and 45 Hz, and a secondary pitch peak at approximately 95 Hz (Fig 3). The sound was generated from a single hit on a percussion instrument (gran cassa), which generated a sound burst with a duration of 500 milliseconds. Each sound burst was separated by intervals generated by a random number generator producing numbers between 1-10. Each digit had an equivalent of 250 milliseconds; so that number 1 represented 250 milliseconds, number 2 represented 500 milliseconds, number 3 represented 750 milliseconds, and so on. These numbers were used to determine the intervals between each sound onset throughout the trial. The track was produced by arranging sound bursts separated by the random intervals until one minute of material was generated. This first minute of material was repeated four more times, but each of these five identical segments was set to a different tempo; the first minute played at 120 bpm, the second at 110, the third at 115, the fourth at 125 and the fifth 130. This 5-minute sequence was then copied and pasted 5 times which then, given the variations in tempo, amounted to 30 minutes and 49 seconds. Based on this method, 30 minutes and 49 seconds soundtrack was produced leaving a 1-second gap at the beginning of the track. A gate processing was inserted in the track to shorten the decay of the gran cassa sound, which had a long vibrating effect. The gate was set at -18.8db threshold, with an attack setting of 1.0 milliseconds, a hold setting of 1 millisecond, and a release of 120 milliseconds. The gran cassa sound was produced hitting a Laurin Drums electronic drum pad triggering a Roland TD-20 Percussion sound module, and normalized to -1 DB. The recording and sound editing was done with the software Cubase Studio 5.

**Fig 3:** Stimulus peak frequencies. Sound administered as stimulation to group two comprised of randomly intermittent sounds consisting of complex wave gamma-range noise with pitch peaks at approximately 33 Hz and 45 Hz, and a secondary pitch peak at approximately 95 Hz.

### Assessments and outcome measures

The baseline visit was completed 1-7 days prior to the start of the intervention and included self-report questionnaires assessing fibromyalgia symptoms (Revised Fibromyalgia Impact Questionnaire) [44], pain severity and interference (Brief Pain Inventory – Short Form) [45], sleep quality (Pittsburgh Sleep Quality Index) [46], depression symptoms (Patient Health Questionnaire PHQ-9) [47], and quality of life (Quality of Life Enjoyment and Satisfaction – Short Form) [48]. The post-intervention visit was completed within 1-7 days of completion of the last treatment session and assessed outcome changes from baseline, as well as measures of patient global impression of change (Patient Global Improvement Impression; PGI-I, and adapted Glasgow Benefit Inventory; GBI) [49,50]. Data from the 11-point Likert scale assessing daily pain levels before and after each session, as recorded by participants in the treatment logs, was also analyzed.

The primary outcome measure of the study was the Revised Fibromyalgia Impact Questionnaire (FIQ) [44], which is a commonly used instrument to evaluate fibromyalgia symptoms. This self-report questionnaire consists of 21 items assessing physical functioning, fibromyalgia symptoms (e.g., pain, stiffness, and fatigue), and overall well-being. Each item of the FIQ questionnaire is based on a 10-point scale, with total scores ranging from 0 to 100, with higher scores indicating worse symptoms. Treatment response was deemed to occur if there was at least a 14% change in the FIQ total score from baseline, in line with the minimal clinically important difference determined by Bennett et al. [51].

The secondary outcome measures consisted of assessments of pain severity and interference using the Brief Pain Inventory - Short Form (BPI-SF) [45]. The BPI-SF is a 9 item self-report questionnaire based on a 10-point scale which is used to evaluate pain severity and the interference of pain on patients’ daily functioning. Pain severity scores are based on the average pain intensity ratings on four items (worst pain, least pain, average pain, pain right now), and each item is rated from 0 (no pain) to 10 (extreme pain), with scores ranging from 0 to 40. Pain interference scores correspond to the average ratings on seven sub-items (general activity, mood, walking ability, normal walk, relations with other people, sleep, and enjoyment of life), and each item is rated from 0 (does not interfere) to 10 (complete interferes), with a range from 0 to 70 [52]. Sleep quality was assessed using the Pittsburgh Sleep Quality Index (PSQI) [46], a self-report questionnaire consisting of 19 items assessing sleep quality and disturbances over a 1-month time interval. The PSQI total score reflects seven different components (sleep quality, sleep latency, sleep duration, habitual sleep efficiency, sleep disturbances, use of medication, and daytime dysfunction), and ranges from 0 to 21, with higher scores indicating worse sleep quality. The Patient Health Questionnaire (PHQ-9) [47] is the 9-item depression module of the Patient Health Questionnaire and is used to assess depression severity over a 2-week time frame, with each item rated from 0 (not at all) to 3 (nearly every day), and total scores ranging from 0 to 27. Lastly, quality of life was assessed using the Quality of Life Enjoyment and Satisfaction (QLES-Q Short Form) [48], a self-report questionnaire with 16 items assessing domains such as physical health, leisure activities, social relationships, general activities, satisfaction with medications and life satisfaction. Each item is scored on a 5-point scale, with total scores ranging from 14 to 70, and higher scores indicating better enjoyment and satisfaction with life [53].

### Randomization

Eligible participants were randomly allocated to one of the study groups (1:1) using a computer-generated randomization list. To assure blinding for participants and the assessor, an independent investigator held the randomization list and performed the patient allocation after the baseline assessment. Patients were encouraged not to disclose any information about the stimulation received to the assessor; however, approximately 15% of patients occasionally volunteered information regarding allocation during the post-intervention visit. After the final visit, all participants were given the opportunity to undertake the treatment offered to the other group.

### Statistical analysis

Data analysis was completed based on intention-to-treat and data collected from all participants enrolled in the study was included in the analysis. For dichotomous outcomes, missing values from post-intervention assessments of individuals who discontinued the study were handled according to the baseline-observation-carry-forward approach as we assumed no change for those where the outcome was unobserved. For continuous outcomes (e.g. treatment log), intention-to-treat meant that we only retained data from participants for whom the information was available to avoid multiple imputations.

Statistical analyses were performed using SPSS 22.0 (IBM Corp., Armonk, NY, USA). Independent sample t-tests were used to assess group differences in demographic and clinical-related parameters at baseline. We analyzed the effects of the intervention on the outcome measures using a 2×2 factor repeated measures analysis of variance with time (baseline and post-intervention) and group (continuous 40 Hz stimulation vs. intermittent gamma-frequency stimulation) as factors. Significant interactions and within-group comparisons were further explored with paired t-tests. Analysis of daily pain levels before and after each treatment session (self-reported in treatment logs) was performed by averaging the daily ratings to reflect changes on a weekly basis. Changes of average pain ratings over the course of the study were analyzed with a repeated measures ANOVA with time (weeks 1-5) and pain ratings (before/after a session) as within-subject factors, and group (40 Hz continuous vs. intermittent stimulation) and treatment response (responders vs. non-responders) as between-subject factors. For all ANOVAs, data were continuous and normally distributed, with no significant outliers and no evidence of sphericity from the Mauchly’s test or violation of homogeneity of variance from the Levene’s test. We also conducted logistic regression analyses to examine the possible influence of baseline clinical outcome variables on treatment response. The independent variables (i.e., fibromyalgia symptoms, pain severity and interference, depression, quality of life, and sleep quality at baseline) were each entered separately on to the model to probe for indices evaluating prediction of response. The alpha level was set at 5% for all tests. Based on previous studies [38], to determine effect size required (*r* = .95) to obtain sufficient statistical power (80%) with the significance level of α = 0.05, the minimum sample size for each group is 20 patients.

## Results

### Patient characteristics

A total of 84 patients were screened for eligibility. Of the patients screened, 4 declined participation and 30 did not meet inclusion criteria for reasons such as recent injury, surgery, and unstable medical conditions, totaling 50 patients enrolled in the study (Fig 1). Of the patients included in the study, 25 were randomized to the continuous 40 Hz vibrotactile RSS group (Group 1), while the other 25 patients were allocated to the intermittent gamma frequency sensory vibrotactile stimulation group (Group 2). Twelve patients withdrew from the study; three participants in Group 1 and nine in Group 2. Of these participants, two reported that the reason for discontinuation of the intervention was related to hypersensitivity or intolerance to the sensory stimulation, whereas the other ten participants reported non-adverse related events, including family issues, traveling, car accident, and difficulties operating the treatment device. Thirty-eight participants of the total sample (76%) completed all study visits.

Demographic and clinical characteristics at baseline are displayed in Table 1. The average age of participants was 50 years (*SD* = 12.27 years), ranging from 22 to 68 years of age. The majority of participants were female (92%) and the average duration of symptoms was 7.9 years (*SD* = 7.1 years). There were no significant baseline differences for socio-demographic or clinical-related parameters between treatment groups. The average total score of the Revised Fibromyalgia Impact Questionnaire (FIQ) at baseline for Group 1 was 70 (*SD* = 17) and 63 (*SD* = 15) for Group 2, a non-statistically significant difference (*p* = 0.15). Seventy percent of the patients reported the presence of a concomitant condition, such as anxiety, depression, chronic fatigue syndrome, and temporomandibular joint disorder. For 84% of the participants, usual care involved regular medication intake for pain, and 86% of participants reported generally making use of complementary approaches as part of the pain management treatment, including meditation, listening to music, yoga, mindfulness or relaxation techniques.

**Table 1:** Demographic and clinical characteristics of study participants at baseline.

	Group 1 (*n* = 25)	Group 2 (*n* = 25)	Total (*n* = 50)
Age (years)	50 ± 12.18	50 ± 12.27	50 ± 12.27
Disease duration (years)	8 ± 7.3	7.9 ± 7.1	7.9 ± 7.1
FIQ total score (0 to 100)	70 ± 17	63 ± 15	67 ± 16
Sex (female/male)	23/2	23/2	46/4
Medication for pain (yes/no)	21/4	21/4	42/8
Self-reported comorbidity *n (%)*			
Anxiety	4 (16%)	4 (16%)	8 (16%)
Depression	8 (32%)	1 (4%)	9 (18%)
Chronic Fatigue Syndrome	2 (8%)	5 (20%)	7 (14%)
Temporomandibular joint disorder	2 (8%)	2 (8%)	4 (8%)
Crohn’s disease, colitis	4 (16%)	3 (12%)	7 (14%)

Values are expressed as mean ± standard deviation. Group 1: continuous 40 Hz vibrotactile rhythmic sensory stimuli; Group 2: intermittent gamma frequency rhythmic sensory vibrotactile stimuli.

### Treatment groups

Repeated measure ANOVA analysis revealed that there was a significant main effect of time (baseline, post-intervention visits), indicating significant changes from baseline to post-intervention in measures of fibromyalgia symptoms, pain interference, depression, and sleep quality (Table 2). An analysis of the interaction between changes in the outcome measures from baseline to post-intervention between both groups (time x group interaction) showed that there were no significant differences between groups on any of the outcome measures. Post-hoc analysis revealed that fibromyalgia symptoms, depression severity, and sleep quality improved significantly among patients in both groups. Pain interference changed significantly from baseline only for participants in Group 2 (*p* < .005). Results also indicated that there were no significant changes from baseline in both groups in measures of pain severity and quality of life, as measured with BPI and QLES-Q, respectively.

**Table 2:** Change in outcome measures from baseline to post-intervention by treatment groups.

	Main effect of Time			Time-by-group interaction			Group 1 (*n* = 25)		Group 2 (*n* = 25)	
	*F* value	*p* value	Partial η^2^	*F* value	*p* value	Partial η^2^	Baseline	Post-intervention	Baseline	Post-intervention
FIQ	16.59	.001	.257	1.48	.228	.030	70 ± 17	57 ± 27 ^(^**^)^	63 ± 14	56 ± 20 ^(^*^)^
BPI - Pain Interference	11.03	.002	.190	.588	.447	.012	7 ± 2	6.38 ± 2	6.15 ± 2	5.02 ± 2 ^(^**^)^
BPI - Pain Severity	3.52	.06	.068	.216	.645	.004	6.4 ± 1.5	5.8 ± 2	6 ± 1.75	5.5 ± 2
PHQ-9	12.91	.001	.212	.868	.356	.018	16.5 ± 6.11	13.7 ± 7.45 ^(^*^)^	12.6 ± 4.61	11 ± 5.14 ^(^*^)^
QLES-Q	3.99	.051	.077	.424	.518	.009	37.42 ± 20	43.50 ± 23	43.85 ± 14	47 ± 15
PSQI	12.683	.001	.209	.663	.420	.014	14.68 ± 2.9	12.96 ± 3.6 ^(^*^)^	12.68 ± 3.8	11.60 ± 4.2 ^(^*^)^

Values are expressed as mean ± standard deviation. Main effect of time (baseline vs. post-intervention) and time-by-group-interaction are reported, including partial eta-squared (η^2^) effect sizes. Results are based upon intention-to-treat analyses. Paired sample t-test

* *p* < 0.05

** *p* < 0.005. Group 1: continuous 40 Hz rhythmic sensory vibrotactile stimuli; Group 2: intermittent gamma frequency rhythmic sensory stimuli. FIQ, Revised Fibromyalgia Impact Questionnaire; Pain Interference (Brief Pain Inventory); Pain Severity (Brief Pain Inventory); PHQ-9, Patient Health Questionnaire-9; QLES-Q, Quality of Life Enjoyment and Satisfaction; PSQI, Pittsburgh Sleep Quality Index.

Daily pain ratings (ranging from 0: no pain to 10: extreme pain) before and after each treatment session, as recorded in the treatment logs, were averaged to reflect changes on a weekly basis. Changes of average pain ratings over the course of the study were analyzed with a repeated measures ANOVA with time (weeks 1-5) and pain ratings (before/after a session) as within-subject factors, and group (40 Hz continuous vs. intermittent stimulation) and treatment response (responders vs. non-responders) as between-subject factors. There was a significant main effect of pain ratings (*p* < .005), suggesting that participants generally reported changes in their pain levels immediately after each session compared to their pain prior to the session (Table 3). However, there was no significant main effect of time (*p* = .116) and there were no significant interactions between pain ratings pre/post-session with week (*p* = .53), treatment response (*p* = .48), or intervention group (*p* = .76). These findings indicate that, regardless of intervention group or treatment response, participants generally reported improvements in pain severity after the sessions, and that the effects of the interventions were already observable during the first week of intervention and did not change significantly from week 1 to week 5.

**Table 3:** Average pain level ratings across treatment groups before and after each intervention session for each week of the study.

	Pain level before session	Pain level after session
Week 1	6.5 ± 1.7	5.7 ±1.8 ^(^**^)^
Week 2	6.3 ±1.8	5.5 ± 2 ^(^**^)^
Week 3	6.1 ± 1.7	5.4 ± 2 ^(^**^)^
Week 4	6.2 ± 1.8	5.3 ± 2.3 ^(^**^)^
Week 5	6.0 ± 2	5.1 ± 2.2 ^(^**^)^

Values are expressed as mean ± standard deviation. Pain ratings ranged from 0 (no pain) to 10 (extreme). Analyses was conducted only for completers (*n* = 38). Paired sample t-test

** *p* < 0.005

Regarding patient’s impression of change as measured with the PGI-I, of the 38 patients who completed the final study visit 50% reported feeling no change in fibromyalgia symptoms, while 44% of participants reported feeling better with the intervention, and 6% indicated that symptoms were worse after completing the study. The average benefit score reported by participants on the GBI was +9 (range: -16 to +72), which suggests that participants perceived an overall improvement of approximately 10% in quality of life after the intervention.

### Clinically meaningful change in the primary outcome measure

We were also interested in whether the statistically significant changes in fibromyalgia symptoms after 5 weeks were clinically relevant. The minimal clinically important difference is a clinical threshold that represents a meaningful change in the patient’s management [54,55]. According to Bennet et al. [51], a 14% or more reduction in the FIQ score from baseline to post-intervention is considered a clinically meaningful improvement in the measure. Based on this criterion, 20 participants (40%) across our study sample presented clinically meaningful changes in fibromyalgia symptoms severity. Additionally, treatment responders presented individual changes in FIQ total score ranging from 14.16% to 90% (*M* = 40.53, *SD* = 23.52). There were no significant differences in treatment response between groups. The average reduction in the FIQ score from baseline for patients in Group 1 was 22.43% (*SD* = 30.29), whereas the average change in fibromyalgia symptoms severity from baseline for those in Group 2 was 16.22% (*SD* = 25.35).

Logistic regression analyses were performed to ascertain whether fibromyalgia symptoms, pain severity and interference, depression, quality of life, and sleep quality at baseline would influence treatment response. Of the variables tested, only the model including baseline pain interference was significantly associated with treatment response (χ^2^ (1) = 6.734, *p* = .009), explaining 17% (Nagelkerke *R*^*2*^) of the variance in response. This result thus suggests that pain interference level at baseline show predictive utility of treatment response for RSS interventions (B = -.396, Wald = 5.432, *p* = .020, OR = .673), indicating that higher pain interference pre-treatment reduces the chances of a patient to respond to an RSS intervention.

## Discussion

The present study investigated the effects of gamma frequency rhythmic sensory stimulation (RSS) on fibromyalgia. We were interested in whether rhythmic sensory stimulation would promote significant changes in fibromyalgia and associated symptoms such as pain severity and interference, depression, sleep quality and quality of life, and whether treatment effects would differ between two treatment parameters. To test that, one group of patients received vibrotactile stimulation from a continuous single-frequency sine wave at 40 Hz and isochronous auditory stimulation with a 160 Hz tone amplitude modulated at 40Hz, while the second group received vibrotactile stimulation from randomly intermittent vibrations consisting of complex wave gamma-range noise.

Our findings suggested that there were significant changes from baseline in measures of fibromyalgia symptoms, pain interference levels, depression severity, and sleep quality, however, these improvements did not differ significantly between both groups. Effects were clinically relevant, with effect sizes in the medium-to-large range. These findings corroborate previous studies, such as Naghdi and colleagues [38], which indicated that fibromyalgia symptoms, pain levels, and sleep quality, significantly improved after RSS with low-frequency (40 Hz) vibroacoustic stimuli. Interestingly, we also found a marked reduction in depression severity in both groups, raising the question of whether the observed changes were associated with a general improvement in the patients’ mood or whether RSS affected common underlying features between depression and fibromyalgia [56–59]. The effects on depression, seemingly independent of pain relief, were unexpected, and the effect of RSS on depression outside a chronic pain setting need further evaluation.

Our results also indicated that, while the intervention did not seem to have a significant impact on pain severity, a significant reduction of the level of pain interference in the patients’ functioning was observed, particularly for participants in Group 2. Pain interference scores correspond to the average ratings on seven sub-items, including general activity, mood, walking ability, relations with other people, sleep, and enjoyment of life, thus measuring functional interference from pain. On the other hand, self-reported pain severity scores on the BPI are based on the average pain intensity ratings in the past 24 hours. It is well known, however, that day-to-day fluctuations in pain levels are affected by factors such as poor sleep quality on the night before and attention to pain [60,61]. Thus, the analysis of the daily pain severity reported in the treatment logs before and after each treatment session may provide a clearer picture of the effect of RSS on daily pain severity. Indeed, results indicated that participants generally reported improvements in their pain severity after the RSS treatment sessions, regardless of group allocation. This finding suggests that, while there were some immediate effects on pain relief, these benefits may not have persisted to the point of a clinically meaningful improvement for some patients. This hypothesis is further corroborated by the observation that, although changes on the daily pain ratings were already noticeable during the first week of the study, the level of pain severity did not change significantly from week 1 to week 5, which may be indicative of a ceiling effect.

Regarding treatment effectiveness, individual differences in treatment response were observed. Study results indicated a clinically relevant symptom decrease in fibromyalgia in 40% of participants in the study, whereas 6% of patients reported that symptoms were worse after completing the study. This range of responses suggests that a variety of underlying factors may determine how patients respond to RSS. For instance, our results suggested that pain interference levels at baseline may have a predictive utility in treatment response. Thus, it is possible to speculate that severe functional interference from pain at baseline, as well as other factors such as the location of tender points in relation to the stimulation targets, hypersensitivity to vibratory stimuli and/or humming sounds, stimulation intensity selected by the patients, and comorbidities such as chronic migraine, may be important factors to be considered prior to commencement of the treatment. Larger studies with a more thorough clinical characterization are needed to elucidate the determinants of the individual differences in treatment responses.

Research to date has generally assumed that the rhythmic pattern of the stimuli sequence is an essential stimulation parameter. This notion is based on the premise that the local mechanical stimulation generated by RSS would drive the mechanoreceptors in the body to respond at the same frequency [41,62]. A hypothesis explored in the present study was that stimulation lacking a clear rhythmic pattern would be unable to drive oscillatory resonance (peripherally or at brain level), hence differences in treatment response between treatment parameters (gamma range RSS vs. complex wave RSS) could indicate potentially distinct underlying mechanisms. However, we found no significant difference in outcomes between groups. One possible explanation for this result is that the parameters of the random and intermittent stimuli presented for one of the experimental groups still preserved a periodical signal that could have driven oscillatory resonance. This interpretation can be further tested by including a sham stimulation. Alternatively, it may be that the stimuli used in the presented study relied on the similar mechanisms of action.

There is no consensus regarding the mechanisms underlying the effects of sensory stimulation on pain. One hypothesis is that the analgesic effect of vibratory stimulation is due to modulation of processes that occur at the spinal cord level [63,64]. According to this view, vibratory stimulation to the skin triggers low-threshold mechanoreceptors, such as Pacinian corpuscles, that inhibit the activity of dorsal horn neurons responsible for transmitting the information about the pain stimulus to the brain [65–72]. In other words, vibratory stimulation inhibits pain by activating inhibitory interneurons in the spinal cord. Another hypothesis suggests that directing attention away from a noxious stimulus also reduces the perception of pain [25]. Cognitive modulation of pain has been rigorously demonstrated by several lines of inquiry [73–77]. It has been shown, for instance, that pain-related activity in brain regions, such as the somatosensory cortices and anterior insula, can be attenuated by cognitive engagement [75].

However, another hypothesis may be postulated in light of recent evidence regarding neural entrainment. There is a growing body of research showing that brain oscillations can be induced by directly stimulating neuronal elements with rhythmic protocols either through sensory input pathways or by using transcranial stimulation techniques that stimulate the brain directly bypassing sensory input [39]. Studies have consistently shown that the presentation of rhythmic visual stimuli (e.g., flickering light) induces phase-locking of brain oscillations in occipital areas at the same frequency of the stimuli and improves the perception of targets presented in phase with the rhythmic stimuli [78–80]. This entrainment effect has also been reported with auditory rhythmic stimuli [81–83] and somatosensory stimuli [84], showing that RSS at frequencies of intrinsic brain-rhythms may be used to induce brain oscillations in a controlled and functionally meaningful way [39,62]. Moreover, a recent study [85] successfully demonstrated that non-invasive light-flicker treatment at 40 Hz resulted in a significant reduction of Aβ peptides in the primary visual cortex of multiple mouse models and induced gene expression associated with morphological changes of microglia, suggesting that 40 Hz gamma oscillations may induce neuroprotective responses in the brain. Thus, it is possible that acoustic-driven rhythmic sensory stimuli may induce neural entrainment, serving as a potential underlying mechanism for the effects of vibratory rhythmic stimulation [62]. Indeed, there is evidence that fibromyalgia is associated with decreased functional connectivity of the pain network in the brain [86,87], including abnormal oscillatory properties of thalamic neurons that are intrinsic 40 Hz oscillators (i.e., thalamocortical dysrhythmia) [88–92]. This hypothesis warrants further investigation to examine whether RSS with gamma-frequency vibroacoustic stimuli indeed drives brain oscillations and may serve to regulate dysrhythmias and enhance connectivity, thus leading to improvements in fibromyalgia symptomatology.

### Limitations

Future studies are needed to confirm the present results. One of the limitations of the current design is the absence of a control condition. Given the high placebo effects shown in previous research [36], it is not possible to rule out that the outcome changes here reported are due merely to the passing of time, placebo effects, or to a Hawthorne effect. Other factors that may have interfered indirectly with the study results is relating to the concurrent or distracting activities participants could have undertaken during the treatment sessions and the possibility of adjustment of the stimulation intensity. We attempted to account for the possibility that participants would undertake other activities during the self-guided sessions by asking participants to record these activities in the treatment log (e.g. browsing the internet, reading, meditation). However, the lack of consistency in the recording of the data prevented an analysis of the type and frequency of these activities, and whether they could have interacted with the effects of the intervention. Participants were given guidelines and recommendations regarding the stimulation intensities. However, considering that fibromyalgia patients often experience symptoms such as hypersensibility to sounds, touch, and vibrations, we allowed for adjustments in the intensity of the stimulation if needed. According to the data recorded in the treatment logs, the vast majority of participants tended to follow the intervention guidelines throughout the sessions. However, it is possible that changes in the stimulation intensity could have interacted with treatment response.

## Conclusions

This study investigated the effects of gamma-frequency rhythmic sensory stimulation on fibromyalgia. We were interested in whether rhythmic sensory stimulation would promote significant changes in fibromyalgia and associated symptoms, and whether treatment effects would differ between two distinct treatment parameters. Our results indicated that there were statistically significant changes from baseline in measures of fibromyalgia symptoms, pain interference, depression, and sleep quality. However, no significant between-group differences were observed. These preliminary findings suggest that gamma-frequency rhythmic sensory stimulation may decrease fibromyalgia symptoms and ease associated comorbidities, such as sleep disturbances and depression. Further research is needed to confirm the present results and to better elucidate the possible mechanisms underlying clinical responses to rhythmic sensory stimulation.

## Supporting information

S1 File Consort checklist. (PDF)

S2 File Research proposal. (PDF)

## References

[1] ClauwDJ. Fibromyalgia: A clinical review. JAMA - J Am Med Assoc. American Medical Association; 2014;311: 1547–1555. 10.1001/jama.2014.3266 24737367

[2] WilliamsDA, GracelyRH. Biology and therapy of fibromyalgia. Functional magnetic resonance imaging findings in fibromyalgia. Arthritis Res Ther. BioMed Central; 2006;8: 224 10.1186/ar2094 17254318PMC1794529

[3] WolfeF, AndersonJ, HarknessD, BennettRM, CaroXJ, GoldenbergDL, et al A prospective, longitudinal, multicenter study of service utilization and costs in fibromyalgia. Arthritis Rheum. Wiley-Blackwell; 1997;40: 1560–1570. 10.1002/1529-0131(199709)40:9<1560::AID-ART4>3.0.CO;2-7 9324009

[4] WolfeF, RossK, AndersonJ, RussellIJ, HebertL. The prevalence and characteristics of fibromyalgia in the general population. Arthritis Rheum. Wiley-Blackwell; 1995;38: 19–28. 10.1002/art.1780380104 7818567

[5] SprottH. What can rehabilitation interventions achieve in patients with primary fibromyalgia? Curr Opin Rheumatol. 2003;15: 145–150. 10.1097/00002281-200303000-00011 12598803

[6] PenrodJR, BernatskyS, AdamV, BaronM, DayanN, DobkinPL. Health services costs and their determinants in women with fibromyalgia. J Rheumatol. The Journal of Rheumatology; 2004;31: 1391–1398. Available: http://www.ncbi.nlm.nih.gov/pubmed/15229962 15229962

[7] CroffordLJ. Meta-analysis of antidepressants in fibromyalgia. Curr Rheumatol Rep. Current Medicine Group; 2001;3: 115 10.1007/s11926-001-0013-611286666

[8] RobinsonRL, JonesML. In search of pharmacoeconomic evaluations for fibromyalgia treatments: a review. Expert Opin Pharmacother. Taylor & Francis; 2006;7: 1027–1039. 10.1517/14656566.7.8.1027 16722813

[9] ArnoldLM, KeckPE, WelgeJA. Antidepressant Treatment of Fibromyalgia: A Meta-Analysis and Review. Psychosomatics. Elsevier; 2000;41: 104–113. 10.1176/appi.psy.41.2.104 10749947

[10] NöllerV, SprottH. Prospective Epidemiological Observations on the Course of the Disease in Fibromyalgia Patients. J Negat Results Biomed. BioMed Central; 2003;6: 10–12. 10.1186/1477-5751-2-4PMC19477512969513

[11] LautenschlägerJ. Present state of medication therapy in fibromyalgia syndrome. Scand J Rheumatol Suppl. Taylor & Francis; 2000;113: 32–6. 10.1080/030097400446616 11028829

[12] HäuserW, ThiemeK, TurkDC. Guidelines on the management of fibromyalgia syndrome - A systematic review. Eur J Pain. Wiley-Blackwell; 2010;14: 5–10. 10.1016/j.ejpain.2009.01.006 19264521

[13] WilkeWS. Treatment of "resistant" fibromyalgia. Rheum Dis Clin North Am. 1995;21: 247–60. Available: http://www.ncbi.nlm.nih.gov/pubmed/7732172 7732172

[14] McNicolE, Horowicz-MehlerN, FiskRA, BennettK, Gialeli-GoudasM, ChewPW, et al Management of opioid side effects in cancer-related and chronic noncancer pain: a systematic review. J Pain. Elsevier; 2003;4: 231–56. 10.1016/S1526-5900(03)00556-X 14622694

[15] NicassioPM, SchumanC, KimJ, CordovaA, WeismanMH. Psychosocial factors associated with complementary treatment use in fibromyalgia. J Rheumatol. 1997;24: 2008–13. Available: http://www.ncbi.nlm.nih.gov/pubmed/9330946 9330946

[16] Wahner-RoedlerDL, ElkinPL, VincentA, ThompsonJM, OhTH, LoehrerLL, et al Use of Complementary and Alternative Medical Therapies by Patients Referred to a Fibromyalgia Treatment Program at a Tertiary Care Center. Mayo Clin Proc. Elsevier; 2005;80: 55–60. 10.1016/S0025-6196(11)62958-3 15667030

[17] BaranowskyJ, KloseP, MusialF, HaeuserW, DobosG, LanghorstJ. Qualitative systemic review of randomized controlled trials on complementary and alternative medicine treatments in fibromyalgia. Rheumatol Int. 2009;30: 1–21. 10.1007/s00296-009-0977-5 19672601

[18] Pioro-BoissetM, EsdaileJM, FitzcharlesM-A. Alternative medicine use in fibromyalgia syndrome. Arthritis Rheum. Wiley-Blackwell; 1996;9: 13–17. 10.1002/art.17900901058945108

[19] BarnesPM, BloomB, NahinRL. Complementary and Alternative Medicine Use Among Adults and Children: United States. National Health Statistics Reports. 2008 p. 24 Available: https://stacks.cdc.gov/view/cdc/526619361005

[20] ThomsonP, JonesJ, BrowneM, LeslieSJ. Why people seek complementary and alternative medicine before conventional medical treatment: A population based study. Complement Ther Clin Pract. Churchill Livingstone; 2014;20: 339–346. 10.1016/j.ctcp.2014.07.008 25156988

[21] LundebergT, NordemarR, OttosonD. Pain alleviation by vibratory stimulation. Pain. No longer published by Elsevier; 1984;20: 25–44. 10.1016/0304-3959(84)90808-X 6333660

[22] ZoppiM, VoegelinMR, SignoriniM, ZamponiA. Pain threshold changes by skin vibratory stimulation in healthy subjects. Acta Physiol Scand.; 1991;143: 439–444. 10.1111/j.1748-1716.1991.tb09256.x 1815478

[23] HollinsM, RoyEA, CraneSA. Vibratory antinociception: Effects of vibration amplitude and frequency. J Pain.; 2003;4: 381–391. 10.1016/S1526-5900(03)00714-4 14622680

[24] KakigiR, ShibasakiH. Mechanisms of pain relief by vibration and movement. J Neurol Neurosurg Psychiatry. 1992;55: 282–286. 10.1136/jnnp.55.4.282 1583512PMC489040

[25] HollinsM, McDermottK, HarperD. How does vibration reduce pain? Perception. 2014;43: 70–84. 10.1068/p7637 24689133

[26] HanssonP, EkblomA. Afferent stimulation induced pain relief in acute oro-facial pain and its failure to induce sufficient pain reduction in dental and oral surgery. Pain.; 1984;20: 273–278. 10.1016/0304-3959(84)90016-2 6393002

[27] LobreWD, CallegariBJ, GardnerG, MarshCM, BushAC, DunnWJ. Pain control in orthodontics using a micropulse vibration device: A randomized clinical trial. Angle Orthod. Edward H. Angle Society of Orthodontists; 2016;86: 625–630. 10.2319/072115-492.1 26496680PMC8601487

[28] JingD, XiaoJ, LiX, LiY, ZhaoZ. The effectiveness of vibrational stimulus to accelerate orthodontic tooth movement: A systematic review. BMC Oral Health. BioMed Central; 2017;17: 143 10.1186/s12903-017-0437-7 29195495PMC5709826

[29] SharmaP, CzyzCN, WulcAE. Investigating the efficacy of vibration anesthesia to reduce pain from cosmetic botulinum toxin injections. Aesthetic Surg J. Oxford University Press; 2011;31: 966–971. 10.1177/1090820X11422809 22001341

[30] CercielloS, RossiS, VisonaE, CoronaK, OlivaF. Clinical applications of vibration therapy in orthopaedic practice. Muscles Ligaments Tendons J. CIC Edizioni Internazionali; 2016;6: 147–156. 10.11138/mltj/2016.6.1.147 27331044PMC4915454

[31] CochraneDJ. Effectiveness of using wearable vibration therapy to alleviate muscle soreness. Eur J Appl Physiol. Springer Berlin Heidelberg; 2017;117: 501–509. 10.1007/s00421-017-3551-y 28168554

[32] VeqarZ, ImtiyazS. Vibration Therapy in Management of Delayed Onset Muscle Soreness. J Clin Diagn Res. JCDR Research & Publications Private Limited; 2014;8: LE01–4. 10.7860/JCDR/2014/7323.4434 25121012PMC4127040

[33] MuceliS, FarinaD, KirkesolaG, KatchF, FallaD. Reduced force steadiness in women with neck pain and the effect of short term vibration. J Electromyogr Kinesiol. Elsevier; 2011;21: 283–290. 10.1016/j.jelekin.2010.11.011 21195628

[34] LurieRC, CiminoSR, GregoryDE, BrownSHM. The effect of short duration low back vibration on pain developed during prolonged standing. Appl Ergon. Elsevier; 2018;67: 246–251. 10.1016/j.apergo.2017.10.007 29122196

[35] RoyEA, HollinsM, MaixnerW. Reduction of TMD pain by high-frequency vibration: A spatial and temporal analysis. Pain.; 2003;101: 267–274. 10.1016/S0304-3959(02)00332-9 12583869

[36] WeberA, WerneckL, PaivaE, GansP. Effects of Music in Combination with Vibration in Acupuncture Points on the Treatment of Fibromyalgia. J Altern Complement Med. 2015;21: 77–82. 10.1089/acm.2014.0199 25635925

[37] CheskyKS, RussellIJ, LopezY, Kondraske GV. Fibromyalgia tender point pain: a double-blind, placebo-controlled pilot study of music vibration using the Music Vibration Table. J Musculoskelet Pain. 1997;5: 33–52. 10.1300/J094v05n03_04

[38] NaghdiL, AhonenH, MacarioP, BartelL. The Effect of Low-Frequency Sound Stimulation on Patients with Fibromyalgia: A Clinical Study. Pain Res Manag. Hindawi; 2015;20: e21–e27. 10.1155/2015/375174PMC432589625545161

[39] ThutG, SchynsPG, GrossJ. Entrainment of Perceptually Relevant Brain Oscillations by Non-Invasive Rhythmic Stimulation of the Human Brain. Front Psychol. Frontiers; 2011;2: 170 10.3389/fpsyg.2011.00170 21811485PMC3142861

[40] HooperJ. An Introduction to Vibroacoustic Therapy and an Examination of its Place in Music Therapy Practice. Br J Music Ther. 2001;15: 69–77. 10.1177/135945750101500205

[41] PunkanenM, Ala-RuonaE. Contemporary Vibroacoustic Therapy: Perspectives on Clinical Practice, Research, and Training. Music Med. 2012;4: 128–135. 10.1177/1943862112445324

[42] SkilleO, WigramT. The effect of music, vocalisation and vibration on brain and muscle tissue: Studies in vibroacoustic therapy In: TonyWigram, Bruce SaperstonRW, editor. The art and science of music therapy: A handbook. New York, NY: Routledge; 1995 pp. 23–57.

[43] LehikoinenP. The physioacoustic method In: DileoC, WigramT, editors. Music, Vibration, and Health. Cherry Hill, NJ: Jeffrey Books; 1997 pp. 209–215.

[44] BennettRM, FriendR, JonesKD, WardR, HanBK, RossRL. The revised fibromyalgia impact questionnaire (FIQR): Validation and psychometric properties. Arthritis Res Ther. BioMed Central; 2009;11: R120 10.1186/ar2783 19664287PMC2745803

[45] CleelandCS, RyanKM. Pain assessment: global use of the Brief Pain Inventory. Ann Acad Med Singapore. 1994;23: 129–138. 10.1016/0029-7844(94)00457-O 8080219

[46] BuysseDJ, ReynoldsCF, MonkTH, BermanSR, KupferDJ, III CFR, et al The Pittsburgh Sleep Quality Index: a new instrument for psychiatric practice and research. Psychiatry Res. Elsevier; 1989;28: 193–213. 10.1016/0165-1781(89)90047-4 2748771

[47] KroenkeK, SpitzerRL. The PHQ-9: A New Depression Diagnostic and Severity Measure. Psychiatr Ann. SLACK Incorporated; 2002;32: 509–515. 10.3928/0048-5713-20020901-06

[48] EndicottJ, NeeJ, HarrisonW, BlumenthalR. Quality of Life Enjoyment and Satisfaction Questionnaire: a new measure. Psychopharmacol Bull. 1993;29: 321–326. 10.1111/j.1365-2850.2011.01735.x 8290681

[49] GuyW. ECDEU Assessment Manual for Psychopharmacology: Revised ECDEU Assessment Manual. Washington, DC: US Government Printing Office; 1976.

[50] RobinsonK, GatehouseS, BrowningGG. Measuring patient benefit from otorhinolaryngological surgery and therapy Ann Otol Rhinol Laryngol. SAGE PublicationsSage CA: Los Angeles, CA; 1996;105: 415–422. 10.1177/000348949610500601 8638891

[51] BennettRM, BushmakinAG, CappelleriJC, ZlatevaG, SadoskyAB. Minimal clinically important difference in the fibromyalgia impact questionnaire. J Rheumatol. The Journal of Rheumatology; 2009;36: 1304–1311. 10.3899/jrheum.081090 19369473

[52] PoquetN, LinC. The Brief Pain Inventory (BPI). J Physiother. Elsevier; 2016;62: 52 10.1016/j.jphys.2015.07.001 26303366

[53] StevanovicD. Quality of life enjoyment and satisfaction questionnaire - short form for quality of life assessments in clinical practice: A psychometric study. J Psychiatr Ment Health Nurs. Wiley/Blackwell (10.1111); 2011;18: 744–750. 10.1111/j.1365-2850.2011.01735.x 21896118

[54] CopayAG, SubachBR, GlassmanSD, PollyDW, SchulerTC. Understanding the minimum clinically important difference: a review of concepts and methods. Spine J. Elsevier; 2007;7: 541–546. 10.1016/j.spinee.2007.01.008 17448732

[55] JaeschkeR, SingerJ, GuyattGH. Measurement of health status: Ascertaining the minimal clinically important difference. Control Clin Trials. Elsevier; 1989;10: 407–415. 10.1016/0197-2456(89)90005-6 2691207

[56] PaeC-U, LuytenP, MarksDM, HanC, ParkS-H, PatkarAA, et al The relationship between fibromyalgia and major depressive disorder: a comprehensive review. Curr Med Res Opin. Taylor & Francis; 2008;24: 2359–2371. 10.1185/03007990802288338 18606054

[57] GracelyRH, CekoM, BushnellMC. Fibromyalgia and depression. Pain Res Treat. Hindawi Limited; 2012;2012: 486590 10.1155/2012/486590 22191023PMC3236322

[58] AgugliaA, SalviV, MainaG, RossettoI, AgugliaE. Fibromyalgia syndrome and depressive symptoms: Comorbidity and clinical correlates. J Affect Disord. Elsevier; 2011;128: 262–266. 10.1016/j.jad.2010.07.004 20674985

[59] ChangMH, HsuJW, HuangKL, SuTP, BaiYM, LiCT, et al Bidirectional Association between Depression and Fibromyalgia Syndrome: A Nationwide Longitudinal Study. J Pain. Churchill Livingstone; 2015;16: 895–902. 10.1016/j.jpain.2015.06.004 26117813

[60] AffleckG, UrrowsS, TennenH, HigginsP, AbelesM. Sequential daily relations of sleep, pain intensity, and attention to pain among women with fibromyalgia. Pain. No longer published by Elsevier; 1996;68: 363–368. 10.1016/S0304-3959(96)03226-5 9121825

[61] LewandowskiAS, PalermoTM, MotteSD la, FuR. Temporal daily associations between pain and sleep in adolescents with chronic pain versus healthy adolescents. Pain. No longer published by Elsevier; 2010;151: 220–225. 10.1016/j.pain.2010.07.016 20719433PMC2939216

[62] BartelLR, ChenREW, AlainC, RossB. Vibroacoustic Stimulation and Brain Oscillation: From Basic Research to Clinical Application. Music Med. 2017;9: 153–166. Available: https://mmd.iammonline.com/index.php/musmed/article/view/542

[63] MeyersonBA, LinderothB. Mechanisms of spinal cord stimulation in neuropathic pain. Neurol Res. 2000;22: 285–292. 10.1080/01616412.2000.11740672 10769822

[64] MoayediM, DavisKD. Theories of pain: from specificity to gate control. J Neurophysiol. 2013;109: 5–12. 10.1152/jn.00457.2012 23034364

[65] HollinsM, CorsiC, SloanP. Pacinian Signals Determine the Direction and Magnitude of the Effect of Vibration on Pain. Perception. 2017;46: 987–999. 10.1177/0301006617694630 28715995

[66] MelzackR, WallPD. Pain Mechanisms: a new theory. Science (80-). 1965;150: 971.532081610.1126/science.150.3699.971

[67] MendellLM. Constructing and deconstructing the gate theory of pain. Pain. No longer published by Elsevier; 2014;155: 210–216. 10.1016/j.pain.2013.12.010 24334188PMC4009371

[68] TorsneyC, MacDermottAB. Disinhibition Opens the Gate to Pathological Pain Signaling in Superficial Neurokinin 1 Receptor-Expressing Neurons in Rat Spinal Cord. J Neurosci. 2006;26: 1833–1843. 10.1523/JNEUROSCI.4584-05.2006 16467532PMC6793628

[69] ToddAJ. Neuronal circuitry for pain processing in the dorsal horn. Nat Rev Neurosci. 2010;11: 823–836. 10.1038/nrn2947 21068766PMC3277941

[70] LuY, DongH, GaoY, GongY, RenY, GuN, et al A feed-forward spinal cord glycinergic neural circuit gates mechanical allodynia. J Clin Invest. American Society for Clinical Investigation; 2013;123: 4050–4062. 10.1172/JCI70026 23979158PMC4381282

[71] DuanB, ChengL, BouraneS, BritzO, PadillaC, Garcia-CampmanyL, et al Identification of spinal circuits transmitting and gating mechanical pain. Cell. Cell Press; 2014;159: 1417–1432. 10.1016/j.cell.2014.11.003 25467445PMC4258511

[72] PeirsC, WilliamsSPG, ZhaoX, WalshCE, GedeonJY, CagleNE, et al Dorsal Horn Circuits for Persistent Mechanical Pain. Neuron. Cell Press; 2015;87: 797–812. 10.1016/j.neuron.2015.07.029 26291162PMC4562334

[73] LeungRH, StromanPW. Neural Correlates of Cognitive Modulation of Pain Perception in the Human Brainstem and Cervical Spinal Cord using Functional Magnetic Resonance Imaging: A Review. Crit Rev Biomed Eng. Begel House Inc.; 2016;44: 33–45. 10.1615/CritRevBiomedEng.2016016540 27652450

[74] VillemureC, BushnellMC. Cognitive modulation of pain: How do attention and emotion influence pain processing? Pain. 2002;95: 195–199. 10.1016/S0304-3959(02)00007-6 11839418

[75] SeminowiczDA, MikulisDJ, DavisKD. Cognitive modulation of pain-related brain responses depends on behavioral strategy. Pain. 2004;112: 48–58. 10.1016/j.pain.2004.07.027 15494184

[76] RoyM, PicheM, ChenJ-I, PeretzI, RainvilleP. Cerebral and spinal modulation of pain by emotions. Proc Natl Acad Sci. 2009;106: 20900–20905. 10.1073/pnas.0904706106 19926861PMC2779826

[77] OssipovMH, DussorGO, PorrecaF. Central modulation of pain. J Clin Invest. American Society for Clinical Investigation; 2010;120: 3779–3787. 10.1172/JCI43766 21041960PMC2964993

[78] de GraafTA, GrossJ, PatersonG, RuschT, SackAT, ThutG. Alpha-Band Rhythms in Visual Task Performance: Phase-Locking by Rhythmic Sensory Stimulation. de LangeFP, editor. PLoS One. Public Library of Science; 2013;8: e60035 10.1371/journal.pone.0060035 23555873PMC3612058

[79] SpaakE, de LangeFP, JensenO. Local Entrainment of Alpha Oscillations by Visual Stimuli Causes Cyclic Modulation of Perception. J Neurosci. Society for Neuroscience; 2014;34: 3536–3544. 10.1523/JNEUROSCI.4385-13.2014 24599454PMC6608988

[80] NotbohmA, KurthsJ, HerrmannCS. Modification of Brain Oscillations via Rhythmic Light Stimulation Provides Evidence for Entrainment but Not for Superposition of Event-Related Responses. Front Hum Neurosci. Frontiers; 2016;10: 10 10.3389/fnhum.2016.00010 26869898PMC4737907

[81] NozaradanS. Exploring how musical rhythm entrains brain activity with electroencephalogram frequency-tagging. Philos Trans R Soc B Biol Sci. The Royal Society; 2014;369: 20130393 10.1098/rstb.2013.0393 25385771PMC4240960

[82] ten OeverS, SchroederCE, PoeppelD, van AtteveldtN, MehtaAD, MégevandP, et al Low-frequency cortical oscillations entrain to sub-threshold rhythmic auditory stimuli. J Neurosci. Society for Neuroscience; 2017;37: 3658–16. 10.1523/JNEUROSCI.3658-16.2017 28411273PMC5426181

[83] HenryMJ, HerrmannB, ObleserJ. Entrained neural oscillations in multiple frequency bands comodulate behavior. Proc Natl Acad Sci. National Academy of Sciences; 2014;111: 14935–14940. 10.1073/pnas.1408741111 25267634PMC4205645

[84] RossB, JamaliS, MiyazakiT, FujiokaT. Synchronization of beta and gamma oscillations in the somatosensory evoked neuromagnetic steady-state response. Exp Neurol. Academic Press; 2013;245: 40–51. 10.1016/j.expneurol.2012.08.019 22955055

[85] IaccarinoHF, SingerAC, MartorellAJ, RudenkoA, GaoF, GillinghamTZ, et al Gamma frequency entrainment attenuates amyloid load and modifies microglia. Nature. Nature Publishing Group; 2016;540: 230–235. 10.1038/nature20587 27929004PMC5656389

[86] CagnieB, CoppietersI, DeneckerS, SixJ, DanneelsL, MeeusM. Central sensitization in fibromyalgia? A systematic review on structural and functional brain MRI. Semin Arthritis Rheum. 2014;44: 68–75. 10.1016/j.semarthrit.2014.01.001 24508406

[87] CifreI, SitgesC, FraimanD, MuñozMÁ, BalenzuelaP, González-RoldánA, et al Disrupted functional connectivity of the pain network in fibromyalgia. Psychosom Med. 2012;74: 55–62. 10.1097/PSY.0b013e3182408f04 22210242

[88] LlinasRR, RibaryU, JeanmonodD, KronbergE, MitraPP. Thalamocortical dysrhythmia: A neurological and neuropsychiatric syndrome characterized by magnetoencephalography. Proc Natl Acad Sci. National Academy of Sciences; 1999;96: 15222–15227. 10.1073/pnas.96.26.15222 10611366PMC24801

[89] LlinásR, RibaryU, JeanmonodD, CancroR, KronbergE, SchulmanJ, et al Thalamocortical dysrhythmia I. Functional and imaging aspects. Thalamus Relat Syst. No longer published by Elsevier; 2001;1: 237–244. 10.1016/S1472-9288(01)00023-1

[90] LlinásR, UrbanoFJ, LeznikE, RamírezRR, Van MarleHJF. Rhythmic and dysrhythmic thalamocortical dynamics: GABA systems and the edge effect. Trends Neurosci. Elsevier Current Trends; 2005;28: 325–333. 10.1016/j.tins.2005.04.006 15927689

[91] SchulmanJJ, CancroR, LoweS, LuF, WaltonKD, LlinásRR. Imaging of Thalamocortical Dysrhythmia in Neuropsychiatry. Front Hum Neurosci. Frontiers; 2011;5: 69 10.3389/fnhum.2011.00069 21863138PMC3149146

[92] RibaryU, IoannidesAA, SinghKD, HassonR, BoltonJP, LadoF, et al Magnetic field tomography of coherent thalamocortical 40-Hz oscillations in humans. Proc Natl Acad Sci. National Academy of Sciences; 1991;88: 11037–11041. 10.1073/pnas.88.24.11037 1763020PMC53068

